# Long non-coding RNA nuclear enriched abundant transcript 1 (NEAT1) modulates inhibitor of DNA binding 1 (ID1) to facilitate papillary thyroid carcinoma development by sponging microRNA-524-5p

This article has been retracted.

**DOI:** 10.1080/21655979.2022.2076498

**Published:** 2022-05-30

**Authors:** Guansheng Liao, Zhuoya Huang, Tianyu Gan, Cong Wu, Xiaolong Wang, Dexiang Li

**Affiliations:** a Department of Thyroid Surgery, Huizhou Central People’s Hospital, Huizhou, Guangdong, China; b Department of Pathology, Huizhou Central People’s Hospital, Huizhou, Guangdong, China

**Keywords:** lncRNA NEAT1, miR-524-5p, *ID1*, papillary thyroid carcinoma

## Abstract

Long non-coding RNA (lncRNA) nuclear-enriched abundant transcript 1 (NEAT1) exerts a pro-oncogenic role in several cancers, whereas its underlying regulatory mechanism in papillary thyroid carcinoma (PTC) progression remains unknown. This research mainly explored the roles of NEAT1 in PTC development. Quantitative real-time polymerase-chain reaction (qRT-PCR) was applied to measure NEAT1, miR-524-5p, and inhibitor of DNA binding 1 (ID1) expression in PTC tissues and cells. Western blot was conducted for detecting the protein levels. MTT, transwell, and flow cytometry assays were applied to assess cell proliferation, metastasis, and apoptosis in PTC cells *in vitro*. The PTC xenograft tumor model was used for investigating the role of NEAT1 *in vivo*. Dual-luciferase reporter assay was utilized for confirming the interaction between miR-524-5p and NEAT1 or ID1. In PTC tissues and cells, NEAT1 was significantly up-regulated. NEAT1 silencing blocked cell proliferation, metastasis, and facilitated apoptosis *in vitro* and impeded xenograft tumor growth *in vivo*. Bioinformatics prediction revealed the existence of binding sites between NEAT1 and miR-524-5p. Besides, ID1 was confirmed as a direct target to miR-524-5p, and the enhancement of ID1 reversed the regulation of miR-524-5p upregulation on cell progression. In addition, NEAT1 promoted PTC development by regulating ID1 expression via sponging miR-524-5p in PTC. In summary, we demonstrate that NEAT1 advanced the process of PTC by miR-524-5p/ID1 axis, which may enhance our comprehension of PTC pathogenesis.

## Highlights

- NEAT1 is elevated in PTC.
- NEAT1 knockdown blocks PTC development in vitro and in vivo.
- NEAT1 directly targets the miR-524-5p/ID1 axis in PTC.

## Introduction

Thyroid carcinoma (TC) is a prevalent endocrine malignant tumor, accounting for 2.1% of the latest cancer diagnosis. TC contains several histological subtypes including papillary thyroid carcinoma (PTC) (about 75% of the total), follicular thyroid carcinoma (FTC) (about 15% of the total) and anaplastic thyroid carcinoma (ATC) (about 1% of the total) [1]. The former two are differentiated thyroid carcinoma (DTC), and the latter is undifferentiated thyroid carcinoma (UTC) [2]. Surgery, chemotherapy, and radiotherapy are the conventional approaches for the treatment of TC [3]. However, these treatments have not yet produced desirable effects as radioiodine-refractory thyroid cancers (5–15% of DTC, 50% of metastatic DTC and ATC) have poor outcomes [4]. The high proportion of iodine-refractory PTC warrants further study as theoretical support for PTC therapy.

Long non-coding RNAs (lncRNAs) are an important type of ncRNAs with no or limited protein-coding capacity [5–9]. Many studies have found that dysregulation of lncRNAs occurred frequently in several pathological states, including cancer. Liu *et al*. clarified that lncRNA X–inactive specific transcript served as a competing endogenous RNA (ceRNA) for miR-34a and modulated TC cell proliferation and tumor growth [10]. LncRNA lung cancer-related transcript 1 (LUCAT1) was involved in PTC development via regulating cell-cycle, proliferation, epigenetic modifications [11]. Nuclear enriched abundant transcript 1 (NEAT1) sponged miR-129-5p to regulate KLK7 expression to participate in PTC development [12]. NEAT1, a 3.2 kb lncRNA located in human chromosome 11, plays vital roles in multiple human diseases and serves as a tumor-promoting lncRNA in multiple cancers, including TC [13–15]. However, the detailed molecular mechanism of NEAT1 in PTC remains unclear.

Increasing studies have elucidated that NEAT1 widely acts as a ceRNA to decoy target miRNAs and regulate the expression of downstream mRNAs [16,17]. To further exploit the downstream miRNA/mRNA networks targeted by NEAT1, we screened and identified the downstream miRNAs and mRNAs of NEAT1. Numerous publications recognized miR-524-5p as a wide tumor suppressor in various cancers [18,19]. Interestingly, miR-524-5p was predicted to be targeted by NEAT1 through bioinformatics analysis. However, the target relationship between miR-524-5p and NEAT1 in PTC development has not been validated. Accordingly, the inhibitor of DNA binding 1 (ID1) was a potential downstream target of miR-524-5p. It was previously mentioned that the activation of the oncogenic AKT signaling pathway was associated with the upregulation of ID1 in PTC progression [20], revealing that ID1 contributed to PTC development. However, the relationship of ID1 associated with NEAT1/miR-524-5p axis in PTC needs further validation.

In this research, we hypothesized that NEAT1 exerted cancer-promoting effects on PTC and NEAT1 controlled the new miRNA/mRNA networks to mediate PTC development. We investigated the expression of NEAT1 in PTC and testified its relationships with miR-524-5p/ID1 axis, aiming to address the new regulatory mechanism of NEAT1 in PTC and further understand PTC pathogenesis.

## Materials and methods

### Tissues collection

PTC tissue samples (*n* = 30) and the corresponding adjacent normal tissues (*n* = 30) were obtained from patients who diagnosed as human papillary thyroid cancer in Huizhou Central People’s Hospital. All the tissues were frozen at −80°C for further using. All patients provided written informed consent. The study was authorized by the Ethics Committee of Huizhou Central People’s Hospital (2021HZ662). The clinical features of the enrolled patients with PTC and the correlation between the clinical features and NEAT1 expression are summarized in Table 1.

**Table 1.** Relationship between NEAT1 expression and clinicopathologic features of papillary thyroid carcinoma patients

	Characteristics n = 30	NEAT1 expression		*P* value
		Low (*n* = 15)	High (*n* = 15)	
Gender				>0.9999
Female	17	8	9	
Male	13	7	6	
Age (years)				>0.9999
≤50	11	6	5	
>50	19	9	10	
TNM grade				0.0209*
I+ II	11	9	2	
III+IV	19	6	13	
Lymph node metastasis				0.0253*
Positive	17	5	12	
Negative	13	10	3	
Tumor size				0.0025*
≤2 cm	13	11	2	
>2 cm	17	4	13	

TNM, tumor-node-metas-tasis; *P < 0.05.

### RNA extraction and quantitative real-time polymerase chain reaction (qRT-PCR)

After extracting total RNA using Trizol Reagent (Invitrogen, Carlsbad, CA, USA), RNA was subjected to reverse transcription with PrimeScript RT reagent kit (TaKaRa, Dalian, China) with random primers or specific stem-loop RT primers for miR-524-5p. And the quantitative PCR was carried out using SYBR Master Mix (TaKaRa). NEAT1 and *ID1* mRNA levels were normalized by GAPDH and miR-524-5p expression was normalized by U6. The expression of NEAT1, miR-524-5p and *ID1* mRNA were analyzed with the method of 2^−ΔΔCt^. The primer sequences (5’-3’) were listed as follows: NEAT1: (F: CCTAGCATGTTTGACAGGCG, R: TGCCACCTGGAAATAAAGCG); miR-524-5p: (F: GCCTACAAAGGGAAGCAC, R: ATCCAGTGCAGGGTCCGAGG); *ID1*: (F: AAACGTGCTGCTCTACGACA, R: GGAACGCATGCCGCCT); GAPDH: (F: CCCACTCCTCCACCTTTGAC, R: CATACCAGGAAATGAGCTTGACAA); U6: (F: CTCGCTTCGGCAGCACA, R: AACGCTTCACGAATTTGCGT).

### Cellular location assay of NEAT1

The cytoplasmic RNA and nuclear RNA from TPC-1 and NIM cells were extracted using a commercial PARIS kit (Invitrogen) according to the protocol. The expression abundance of NEAT1 in cytoplasm or nucleus was checked by qRT-PCR, with GAPDH as an internal reference in cytoplasm and U6 as an internal reference in nucleus.

### Cell culture and transfection

Human PTC cell lines (IHH-4, TPC-1, and NIM) and human normal thyroid cell line (Nthy-ori 3–1) were purchased from Bio-Vector NTCC Inc. (Beijing, China). The cells were cultivated in DMEM (high glucose; Weike Biotechnology, Shanghai, China) with 10% fetal bovine serum (FBS; Genetimes, Shanghai, China) in an incubator at 37°C with 5% CO_2_. Small interfering RNA (siRNA) antagonizing NEAT1 (si-NEAT1), siRNA against *ID1* (si-*ID1*), miR-524-5p mimics (miR-524-5p), miR-524-5p inhibitor (anti-miR-54-5p), NEAT1-overexpressing vector (NEAT1), *ID1* overexpression plasmid (*ID1*) and their negative controls were obtained from Sangon Biotech (Shanghai, China). The oligonucleotide and vector were introduced into PTC cells by using Lipofectamine 3000 Reagent (Invitrogen).

### MTT assay

To test the viability of TPC-1 and NIM cells, MTT assay was performed. Following 24 h, 48 h, or 72 h incubation, the transfected cells in 96-well plate were incubated with MTT (Solarbio, Beijing, China) for 4 h at 37°C, then the DMSO was added to solubilize the formazan. The absorbance was monitored by a Multiscan Spectrum (Petenov, Beijing, China) at 490 nm.

### Flow cytometry assay

Annexin V-FITC&PI apoptosis detection kit (Solarbio) was used for assessing the apoptosis rate. Following 48 h cultivation, the transfected cells were incubated to label with Annexin V- FITC and PI solution. The apoptosis rate was evaluated by using flow cytometry (Agilent, Beijing, China).

### Transwell assay

Transwell chambers with a matrigel matrix (Corning, Tewksbury, MA, USA) were utilized for detecting the invasion capacity of PTC cells. The lower part of the chamber was filled with a complete medium, while the transfected TPC-1 and NIM cells were added into the top chamber supplemented with DMEM without FBS and maintained for 24 h. The cells that invaded to the bottom surface were fixed and stained, then counted using a light microscope.

### Western blot assay

The lysis of cells was administered by RIPA lysis buffer (Solarbio) for extracting proteins. The extracted protein samples were separated by SDS-PAGE and transferred onto a PVDF membrane. Following 3 h blocking in nonfat milk, the membrane was incubated with primary antibodies at 4°C for 12–16 h and then incubated with secondary antibody (HRP-conjugated anti-mouse secondary antibody) for 2 h. An ECL kit (Vazyme, Nanjing, China) was used to detect the chemiluminescence intensity of protein bands. The primary antibodies were Anti-*ID1* (bs-4852 R), anti-CyclinD1 (bs0623R), anti-Bax (bs-0127 R) and anti-MMP9 (bs-0397 R), which were obtained from Bioss (Beijing, China).

### Dual-luciferase reporter assay

Online data base Starbase 3.0 was applied to predict the potential-binding sites between NEAT1 and miR-524-5p, or miR-524-5p and *ID1* 3ʹUTR. Briefly, the wild-type NEAT1 or *ID1* 3ʹUTR that contained the putative miR-524-5p binding sites or a mutant NEAT1 or *ID1* 3ʹUTR sequence was amplified and cloned into psiCHECK2 vector (Promega, Madison, WI, USA) to generate WT-NEAT1, MUT-NEAT1, *ID1* 3ʹUTR-WT, or *ID1* 3ʹUTR-MUT. The luciferase reporter vectors (400 ng) together with 50 nM miR-524-5p or miR-NC and 50 ng renilla luciferase reporter vectors (pRL-TK) were co-introduced into TPC-1 and NIM cells. The luciferase activity was evaluated using a luciferase activity detection kit (Solarbio). Renilla luciferase acted as the normalization factor of firefly luciferase.

### Mice xenograft models

The animal studies were authorized by the Animal Care Committee of Huizhou Central People’s Hospital (HZ2021116). The six-week-old nude mice were obtained from Vital River (Beijing, China), and segmented into two groups as sh-NEAT1 and sh-NC (Genechem, Shanghai, China) group (*n* = 7 per group). The TPC-1 cells (3 × 10^6^ control or NEAT1 knockdown) were injected into nude mice. We detected the volume of tumors by every 4 days for 27 days with the formula: volume (mm^3^) = 1/2 × length × width ^2^. The excised xenograft tumors were then subjected to weight measurement and further analysis.

## Statistical analysis

All the data were performed in at least three independent repetitions and presented as the mean ± standard deviation (SD) using GraphPad Prism 7. Significances of group mean differences were determined by using the unpaired Student’s *t*-test (two-tailed, unequal variances) or one-way ANOVA for multiple comparisons. Statistical significance was considered at *P* < 0.05.

## Results

We hypothesized that NEAT1 exerted the oncogenic effects on PTC by governing the miR-524-5p/*ID1* axis. We testified the expression pattern of NEAT1 in PTC and conducted loss-of-function assays to determine its functions. Moreover, the binding relationship between miR-524-5p and NEAT1 or *ID1* in PTC development was confirmed. These findings aimed to propose a new mechanism regarding NEAT1ʹs functions in PTC.

## NEAT1 was up-regulated in PTC tissues and cells

We first detected NEAT1 expression in PTC tissue samples and cell lines. NEAT1 expression was enhanced in PTC tissue samples relative to adjacent normal tissue samples (Figure 1(a)). As expected, NEAT1 expression was higher in PTC cells (IHH-4, TPC-1, and NIM cells, especially in TPC-1 and NIM cells) than in normal cells (Nthy-ori 3–1 cells) (Figure 1(b)). The cellular location assay displayed that NEAT1 showed a relatively higher expression in cytoplasm relative to nucleus, indicating that NEAT1 was mainly located in the cytoplasm (Figure 1(c,d)). Our data suggested NEAT1 might exert a pro-oncogenic effect on PTC development.

**Figure 1.** NEAT1 was overexpressed in PTC. (a) NEAT1 level in PTC and normal tissues was examined by qRT-PCR. (b) NEAT1 expression was measured via qRT-PCR in PTC cells (IHH-4, TPC-1, and NIM) and human normal thyroid cells (Nthy-ori 3–1). (c and d) The cellular location of NEAT1 in cytoplasm or nucleus of PTC cells was checked. *P < 0.05.

## NEAT1 silencing repressed the proliferation and invasion while promoted apoptosis in TPC-1 and NIM cells

To further explore the functions of NEAT1 in PTC, si-NEAT1 or si-NC was introduced into TPC-1 and NIM cells. The level of NEAT1 expression was dramatically declined in TPC-1 and NIM cells after transfection with si-NEAT1 compared with negative controls (Figure 2(a)). The transfection of si-NEAT1 reduced the cell viability (Figure 2(b,c)) and invasion (Figure 2(e)), but induced apoptosis increased (Figure 2(d)) in si-NEAT1-transfected cells with respect to the negative control. Meanwhile, the effects of si-NEAT1 on viability, invasion, and apoptosis were also verified by the decrease in protein expression in viability-related CyclinD1, invasion-related MMP9, and increase in pro-apoptosis marker Bax in TPC-1 and NIM cells as in contrast to the negative control (Figure 2(f,g)). Taken together, NEAT1 interference restrained the malignant behaviors of PTC cells.

**Figure 2.** NEAT1 knockdown inhibited PTC cell malignant behaviors. PTC cells (TPC-1 and NIM cells) were transfected with or without si-NC or si-NEAT1. (a) NEAT1 expression was measured by qRT-PCR in PTC cells. (b and c) MTT assay was used for measuring cell viability. (d) The apoptosis rate was assessed through flow cytometry in PTC cells. (e) Transwell assay was applied for evaluating the invasion ability in PTC cells. (f and g) The protein expression of CyclinD1, Bax, and MMP9 were detected by western blot in PTC cells. *P < 0.05.

## NEAT1 regulated PTC cell proliferation, invasion, and apoptosis via sponging miR-524-5p

To further seek the potential molecular mechanism of NEAT1 in PTC, StarBase v2.0 was applied to predict the putative targets of NEAT1. The results displayed the existence of binding sites between miR-524-5p and NEAT1 (Figure 3(a)). To verify whether NEAT1 targets to, dual-luciferase reporter assay was carried out. WT-NEAT1 luciferase activity was remarkably inhibited by miR-524-5p, while MUT-NEAT1 luciferase activity had no significant difference (Figure 3(b,c)). In PTC cells, miR-524-5p level was negatively modulated by NEAT1 (Figure 3(d)). In PTC tissues and cells, miR-524-5p was significantly down-regulated (Figure 3(e,f)). In PTC tissue samples, NEAT1 expression was observed to be inversely correlated with miR-524-5p expression (Figure 3(g)). Furthermore, suppressing the level of NEAT1 blocked proliferation and invasion, but facilitated apoptosis, while the effects were reversed by downregulation of miR-524-5p (Figure 3(h–m)). Together, NEAT1 is combined with miR-524-5p to regulate PTC cell behaviors.

**Figure 3.** NEAT1 sponged miR-524-5p. (a) Binding region between miR-524-5p and NEAT1 was predicted by Starbase 2.0. (b and c) The interaction between miR-524-5p and NEAT1 was further verified by dual-luciferase reporter system. (d) The effects of NEAT1 silencing or upregulating on miR-524-5p expression were assessed by qRT-PCR in PTC cells. (e and f) MiR-524-5p expression in PTC or corresponding normal tissues and cells was measured by qRT-PCR. (g) The correlation between the expression of miR-524-5 and NEAT1 was analyzed by Pearson correlation analysis. (h–k) The viability, apoptosis and invasion were assessed via MTT assay, flow cytometry and transwell assay in PTC cells transfected with si-NEAT1 + anti-miR-524-5p or negative control. (l and m) The protein expression levels of CyclinD1, MMP9 and Bax which were the representative markers for proliferation, metastasis and apoptosis were detected by western blot. *P < 0.05.

## MiR-524-5p targeted *ID1* 3ʹUTR

Based on the StarBase v2.0 results, *ID1* was a putative target of miR-524-5p (Figure 4(a)). This putative was further verified by the noticeable decrease in luciferase activity in *ID1* 3ʹUTR-WT in PTC cells introduced with miR-524-5p and dual-luciferase reporter plasmids when compared with negative control (Figure 4(b,c)). In PTC tissues and cells, *ID1* expression was found to be markedly increased (Figure 4(d–g)). Besides, the *ID1* mRNA level correlated negatively with the expression of miR-524-5p (Figure 4(h)). The mRNA and protein level of *ID1* were decreased by miR-524-5p but increased by anti-miR-524-5p (Figure 4(h–l)). These data revealed *ID1* was a target of miR-524-5p.

**Figure 4.** MiR-524-5p targeted *ID1* 3ʹUTR. (a) The sequence of *ID1* 3ʹUTR containing the binding sites for miR-524-5p was exhibited. (b and c) The interaction luciferase between miR-524-5p and *ID1* was verified using dual-luciferase reporter assay. (d and e) The mRNA and protein of *ID1* levels in PTC and normal tissues were detected by qRT-PCR and western blot. (f and g) The mRNA and protein of *ID1* levels in PTC cells (IHH-4, TPC-1 and NIM) and human normal thyroid cells (Nthy-ori 3–1) were detected by qRT-PCR and western blot. (h) The correlation between *ID1* and miR-54-5p was presented by Pearson correlation coefficient. (i–l) *ID1* mRNA and protein levels were measured in TPC-1 and NIM cells after transfection with miR-NC, miR-524-5p, anti-miR-NC, or anti-miR-524-5p by qRT-PCR and western blot. *P < 0.05.

## Upregulation of *ID1* reversed the effects of miR-524-5p overexpression in PTC cells

To further explore the interaction of miR-524-5p and *ID1* in PTC, control, rescue assays were performed. The transfection of *ID1* reversed miR-524-5p overexpression mediated suppression of PTC cell viability (Figure 5(a,b)), and similar results were found in invasion (Figure 5(d)). However, miR-524-5p overexpression-induced apoptosis was mitigated by increasing *ID1* in TPC-1 and NIM cells (Figure 5(c)). Besides, CyclinD1, MMP9, and Bax protein levels also supported the above results in PTC cells (Figure 5(e,f)). Collectively, miR-524-5p exerted the anti-cancer role via inhibiting *ID1* expression in PTC cells.

**Figure 5.** *ID1* counteracted the inhibitory impacts of miR-524-5p on cell proliferation, invasion, and the promotion impact on apoptosis in TPC-1 and NIM cells. The TPC-1 and NIM cells were transfected with control, miR-NC, miR-524-5p, miR-524-5p + pcDNA or miR-524-5p + *ID1*. (a–d) Cell viability, apoptosis rate, and invasive ability were detected. (e and f) CyclinD1, Bax, and MMP9 protein levels were detected by western blot in PTC cells. *P < 0.05.

## NEAT1 sponged miR-524-5p to regulate *ID1* expression

Next, we investigated the relationship among NEATI, miR-524-5p, and *ID1* in TPC-1 and NIM cells, respectively. Western blot results indicated that NEAT1 silencing reduced ID1 protein expression in TPC-1 and NIM cells, while ID1 protein expression in the anti-miR-524-5p + si-NEAT1 group returned to normal (Figure 6(a,b)). These data indicated that the level of ID1 protein was regulated by NEAT1/miR-524-5p pathway.

**Figure 6.** NEAT1 sponged positively miR-524-5p to regulate *ID1* expression. The TPC-1 and NIM cells were transfected with control, miR-NC, miR-524-5p, miR-524-5p + pcDNA or miR-524-5p + NEAT1. (a and b) The protein level of ID1 was detected by western blot. *P < 0.05.

## NEAT1 knockdown suppressed xenograft tumor growth *in vivo*

To further explore the functions of NEAT1 *in vivo*, mice model experiments were constructed. qRT-PCR assay confirmed that stable transfection of sh-NEAT1 efficiently silenced NEAT1 expression in the cancer cells (Figure 7(a)). Compared to the sh-NC group, tumor volume and weight both dramatically decreased in sh-NEAT1 group (Figure 7(b,c)). The expression levels of *ID1* mRNA, *ID1* protein, and NEAT1 were decreased significantly, while miR-524-5p expression was increased (Figure 7(d,e)), which indicated that the knockdown of NEAT1 can upregulate miR-524-5p and downregulate *ID1 in vivo*. These data demonstrated that NEAT1 depletion inhibited xenograft tumor growth *in vivo*.

**Figure 7.** NEAT1 knockdown suppressed xenograft tumor growth *in vivo*. (a) The expression of NEAT1 in TPC-1 cells with sh-NC or sh-NEAT1 transfection. (b and c) The tumor volume and weight were shown. (d) The expression levels of NEAT1, miR-524-5p and *ID1* mRNA were detected. (e) The protein expression of ID1 was measured via western blot. *P < 0.05.

## Discussion

In recent years, the involvement of in the regulation of the cancer processes has become an active area of research. Numerous studies have shown the pivotal roles of lncRNAs in the development of PTC. Wu *et al*. claimed that SNHG15 sponged miR-200a-3p regulate *YAP1-Hippo* expression in PTC [21]. Sun *et al*. revealed that lnc00152 functioned as a cancer promoter in PTC by miR-497/*BDNF* pathway [22]. Feng *et al*. proposed that ASMTL-AS1 suppressed glycolysis and tumor growth via regulation of miR-93-3p/miR-660/*FOXO1* pathway in PTC [23]. In terms of NEAT1, recent research has shown that NEAT1 knockdown led to an inhibition in PTC development through miR-126/NEAT1/*VEGFA* axis [24]. NEAT1 silencing suppressed the radioiodine refractory by governing miR-101-3p/FN1/PI3K-AKT axis in PTC [25]. In addition to PTC, the aberrant overexpression of NEAT1 was also observed in other types of cancer, such as glioma, hepatocellular carcinoma, and laryngeal cancer [16,17,26,27], and the oncogenic effects of NEAT1 on cancer cell proliferation, migration, and invasion were verified. Consistent with the previous findings, herein, NEAT1 was significantly upregulated in PTC cells and tissues. Also, NEAT1 depletion limited the proliferation and invasion but promoted apoptosis of PTC cells, while also restrained xenograft tumor growth *in vivo*. Our results revealed NEAT1 expedited PTC progression, hinting that the target inhibition of NEAT1 might be a promising strategy for PTC therapy in clinical practice.

Furthermore, miR-524-5p was a candidate miRNA sponged by NEAT1, and we further testified the targeting relationship of NEAT1 to miR-524-5p. Several studies have reported that dysregulation of miR-524-5p was related to the development of diverse cancers. MiR-524-5p was downregulated in gastric cancer, and miR-524-5p restoration retarded the proliferation and metastasis, while accelerated the apoptosis of gastric cancer cells *in vitro* [28]. The poor expression of miR-524-5p was also documented in glioma, and miR-524-5p overexpression restrained glioma cell proliferation by targeting *Jagged-1* or *Hes-1 in vitro* [29]. In particular, miR-524-5p was lowly expressed in PTC, and its upregulation retarded PTC development by targeting *FOXE1* and *ITGA3* [30]. Consistently, a decrease of miR-524-5p expression was detected in PTC. The restoration experiments suggested that miR-524-5p deficiency counteracted the inhibition in proliferation and mobility and the enhancement in apoptosis caused by knockdown of NEAT1, indicating that NEAT1 regulated PTC cell biological behaviors by decoying miR-524-5p. We also performed functional assays and displayed that miR-524-5p enrichment repressed PTC cell proliferation and invasion, but enhanced cell apoptosis, exposing the tumor-suppressive role of miR-524-5p in PTC.

Interestingly, miR-524-5p targeted *ID1*, and we ensured that NEAT1 positively modulated *ID1* expression via mediating miR-524-5p. Accumulating evidences indicated that *ID1* was associated with tumor progression through an aberrant change of cell behaviors. For examples, Hu *et al*. demonstrated that the expression level of *ID1* was notably elevated, and the depletion of *ID1* hampered the proliferation and metastasis in penile squamous cell carcinoma cells [31]. Besides, the high expression of *ID1* promoted cell proliferative ability and metastasis, and suppressed apoptosis in salivary adenoid cystic carcinoma cells [32]. Consistent with the results, in our study, *ID1* was highly expressed in PTC tissue specimens and cells. Meanwhile, miR-524-5p upregulation-mediated suppression in proliferation and metastasis and promotion in apoptosis could be reversed by *ID1* overexpression in PTC cells. Taken together, NEAT1 functioned as a cancer promoter by regulating miR-524-5p/*ID1* axis in PTC.

## Conclusion

In summary, NEAT1 was highly expressed in PTC. NEAT1 knockdown resulted in the repression of proliferation, invasion, and the stimulation of apoptosis in PTC cells, indicating that the depletion of NEAT1 might be an effective strategy for PTC treatment. Moreover, NEAT1 promoted the process of PTC via regulating miR-524-5p/*ID1* axis. The novel NEAT1/miR-524-5p/*ID1* regulatory network may provide a new prospect in the mechanism of PTC.

## Supplementary Material

Supplemental Material

## The availability of data and materials

All data generated or analyzed during this study are available from the corresponding author on reasonable request.
